# Survey of Nursing Staff's Training on Early Warning Ability for Inpatients with “Three Infarcts and One Hemorrhage”

This article has been retracted.

**DOI:** 10.1155/2021/3745523

**Published:** 2021-08-16

**Authors:** Zhoumin Shen, Chanjuan Tang, Yanjun Hu, Yimin Cai, Huali Chen, Hongjiao Chen, Yuyu Liu, Nian Xie

**Affiliations:** ^1^Nursing Department, Hunan Provincial People's Hospital, Changsha 410013, Hunan, China; ^2^Department of Respiratory Medicine, Hunan Provincial People's Hospital, Changsha 410013, Hunan, China; ^3^Department of Nursing, Hunan Normal University School, Changsha 410013, Hunan, China

## Abstract

**Methods:**

A total of 787 nursing staff in a tertiary referral center in Changsha City, Hunan Province, were selected using a convenient sampling method. We used an online questionnaire designed by ourselves to survey them. The content of the questionnaire primary included basic information, related knowledge of the nursing staff on the potential risk prediction and precontrol of inpatients with “three infarcts and one hemorrhage,” relevant information on improving early warning scores, management of clinical early warning, training needs, and training methods.

**Results:**

Over 50% of the nursing staff had little understanding about the risk warning knowledge of inpatients with “three infracts and one hemorrhage,” and the degree of understanding was related to education, job title, and working years. The nursing staff with higher education level or professional title or longer working experience have a better understanding of the risk warning knowledge of inpatients with “three infracts and one hemorrhage.”

**Conclusion:**

The cognitive competence of nursing staff in a tertiary referral center in Changsha City, Hunan Province, on the early warning ability of inpatients with “three infarcts and one hemorrhage” needs to be improved. Medical institutions should actively train nursing staff on early warning ability for inpatients with “three infarcts and one hemorrhage” to improve the nursing staff's awareness and patients' safety and efficiency.

## 1. Introduction

Myocardial infarction, pulmonary embolism, cerebral infarction, and dangerous hemorrhage are collectively referred to as “three infarcts and one hemorrhage” in clinical medicine. The condition of hospitalized patients life-threatening at any time with “three infarcts and one hemorrhage” changes rapidly. Prior to the occurrence of accidental death or deterioration of the condition, obvious physiological characteristics usually appear [1, 2]. Therefore, improving the cognition on early warning ability of inpatients is very critical. Nursing risk early warning is the early warning and prevention of existing or potential disease risks in nursing services, and it is an important means of nursing safety management [3–5]. Nurses are direct observers of subtle changes in the patient's condition. They are on the frontline of patient care and generally make a judge of the patients' condition relying on their clinical experience or intuition. Lack of scientific and objective standards may lead to misdiagnosis, missed diagnosis, or delay in treatment [6]. Nursing risk early warning refers to the implementation of dynamic monitoring of the patient's condition during the entire nursing service process, as well as the analysis, early warning, and alarm of all unsafe events such as nursing accidents, nursing complaints, and complications to provide risk prevention and resolution for hospitals so as to ensure the safe and normal operation of hospital nursing work [7].

The purpose of this study is to understand the nursing staff's cognition and training willingness on early warning ability of hospitalized patients. As a result, targeted early warning prevention and control system training will be carried out to improve the ability of early identification and assistance of nurses in the treatment of inpatients with “three infarcts and one hemorrhage,” to ensure patient safety and improvement of nursing quality.

## 2. Method

### 2.1. Survey Object

In this study, a simple random sampling method was adopted to conduct a questionnaire survey on clinical first-line nurses in a tertiary hospital in Changsha City.

  The inclusion criteria include the following: ① all participants who voluntarily agreed to participate in this study and provided written informed consent and ② nurse in the inpatient department of a tertiary hospital
  The exclusion criteria include the following: ① noninpatient department nurses including outpatient department, emergency department, supply room, operating room, endoscopy room, and others and ② nursing staff who are not willing to participate in this study

In the end, a total of 800 questionnaires were issued, and 787 valid questionnaires were recovered, with an effective recovery rate of 98.38%.

### 2.2. Research Tools and Methods

#### 2.2.1. Questionnaire Preparation

This study uses a questionnaire survey method to study the cognition and training willingness of nurses in a tertiary hospital on the early warning ability of inpatients. The content of the questionnaire is set by the researcher on the basis of literature review and expert consultation. In this questionnaire, five sections will be included: ① a general information survey form including gender, education level, professional title, years of work experience, and place of work; ② investigation of the knowledge of medical technicians on the potential risk prediction and precontrol of inpatients with “three infarcts and one hemorrhage”: there are 17 items, divided into single-choice questions and multiple-choice questions; ③ investigation of improved early warning scoring: a total of 10 items are included, which are single-choice questions; ④ survey on the knowledge of clinical early warning management: 7 items are included in the form of single-choice questions and multiple-choice questions; and ⑤ survey on training needs, time, and willingness: 5 items are included in form of single-choice questions.

### 2.3. Reliability and Validity

Forty clinical first-line nurses with the same background as the research subjects were selected for preexperiment, and the reliability coefficients of Cronbach's *α* in part ②③④⑤ of the survey questionnaire were 0.83, 0.74, 0.85, and 0.82, respectively. The content validity of each item (CVI) in the questionnaire conducted by 10 statisticians and clinical nursing experts is 0.80∼1.0. The average CVI of the parts ②③④⑤ is 0.84, 0.83, 0.95, and 0.81, respectively.

### 2.4. Data Processing and Analysis

We used the SPSS 25.0 software to statistically analyze and evaluate all collected data. Descriptive statistical analysis methods such as percentage, mean, and standard deviation were mainly adopted in this work.

## 3. Result

### 3.1. The General Information of Research Object

A total of 787 individuals were selected as research objects for this study. Among them, 86 were males accounting for 10.9%, while the other 701 were females accounting for 89.0%. The selected objects have different educational levels: there were 32 who graduated from junior college (4.1%), 605 undergraduates (76.8%), and 150 who had masters and above level of education (19.1%). From the perspective of professional title, 368 were with junior professional title (accounting for 46.80%). The proportion of intermediate professional title, deputy senior professional title, and senior professional title was 38.9%, 12.2%, and 2.1%, respectively. For years of work experience, the objects who worked for 10–20 years had the maximum proportion which is up to 35.5%. The proportion of working for 5–10 years, 2–5 years, ≤2 years, and >20 years was 30.3%, 13.7%, 10.8%, and 9.5%, respectively. In addition, work location is also one of our investigation factors in this study. The work location of these research objects was mainly distributed in Tianxin Pavilion (47.5%) and Mawangdui (42.6%). The research objects that came from Yuelu Mountain had a very small proportion accounting for 9.6%. The general information of research objects is shown in Figure 1.

### 3.2. Survey on the Current Status of Nurses of Knowledge about Risk Warning of Inpatients with “Three Infarcts and One Hemorrhage”

According to the current status of nurses of understanding of the “three infarcts and one hemorrhage” inpatient risk warning, we conducted investigations and the percentage of each item is recorded in Table 1.

### 3.3. Investigation on the Status of Nurses Came from Different Backgrounds on the Early Warning Ability of Inpatients with “Three Infarcts and One Hemorrhage”

Based on the difference of nurses in gender, education level, professional title, years of work experience, and work location, we studied and concluded the status of selected nurses on the early warning ability of inpatients with “three infarcts and one hemorrhage.” The statistical data are listed in Table 2.

### 3.4. Nursing Staff's Needs for the Early Warning Ability and Related Training of “Three Infarcts and One Hemorrhage” Inpatients

According to the current situation and statistical data analysis of nurses on the early warning ability of inpatients with “three infarcts and one hemorrhage,” we did a questionnaire about nursing staff's needs for cognition and training willingness on early warning ability of inpatients. The results are concluded in Table 3.

## 4. Discussion

### 4.1. The Nurses Have Less Knowledge on Risk Warning for Inpatients with “Three Infarcts and One Hemorrhage,” and the Relevant Training Is Necessary

In Table 1, the results of this survey showed that there were 543 nurses who have received training on the prevention and control of “three infarcts and one hemorrhage,” accounting for 69% of the total. 421 nurses were aware of the Stroke Risk Scorecard and occupied 53.49% of the total number of investigations. And 529 nurses had the experience of the treatment process of pulmonary embolism (67.22%). 100% of nurses believed that it is necessary to train nurses on the knowledge of “three infarcts and one hemorrhage.” In a recent work, Ye and her team members conducted a questionnaire survey on 107 nurses from a local hospital in Zunyi [8]. The score of the knowledge related to predicting and precontrolling the potential risks of inpatients has been collected which is 37.78 ± 10.19, and the results showed that the nurses have a score of ≥60, accounting for only 2.8%. She believed that nurses have little knowledge of potential risk prediction and precontrol of inpatients, which is related to the lack of training and insufficient clinical application of high-risk prediction tools. The early warning system helps to identify changes in the patient's condition so that timely response measures can be taken. Lambert [9] thought that early warning was a useful tool to help alert staff to clinically deteriorating children by periodic observation of physiological parameters, generation of a numeric score, and predetermined criteria for escalating urgent assistance with a clear framework for communication. In addition, the early warning system can also ensure timely identification of patients with potential or established critical illnesses and ensure that skilled staff makes appropriate responses in a timely manner. In Gerry's work, the early warning scoring system has many deficiencies in methodology, when it is used as a predictive model to identify early clinical deterioration of hospital patients [10]. He suggested that future work should follow recommended methods to develop and evaluate early warning scores and investigate the impact and safety of using these scores in clinical practice. Martín-Rodríguez et al. [11], Ye et al. [12], and Rathore et al. [13] found that the high-risk early warning system has a preventive effect on the occurrence of adverse events, improving the quality of care and the management level of critically ill patients and protecting the safety of inpatients. Sutherasan believed that the patients can be classified via an early warning score system according to the disease severity [14]. The occurrence of accidents and complications can be reduced by taking targeted nursing measures and assigning different levels of nurses. Furthermore, the implementation of early warning and nursing intervention can significantly reduce the total length of hospital stay in patients.

### 4.2. Nursing Staff at Different Levels Have Different Cognition on Early Warning Ability of Inpatients with “Three Infarcts and One Hemorrhage”

In this study, we found that nursing staff at different levels have different cognition of the early warning ability of inpatients with “three infarcts and one hemorrhage” from Table 2. The findings showed that the degree of understanding of the risk warning knowledge of inpatients with “three infarcts and one hemorrhage” had a positive correlation with education level, professional title, and working years. Generally speaking, the nurses have a deeper understanding of the risk warning knowledge of inpatients with “three infarctions and one bleeding” with higher education level, higher professional title, or longer working years. These conclusions were consistent with the results of many previous investigations. In some previous works, researchers believed that the early warning ability of high-level nurses was higher than that of low-level nurses. The early warning ability of nurses was affected by many aspects, while the knowledge and training skills related to first aid were the main influencing factors [15–17]. As nurses from different backgrounds have different levels of knowledge of early warning, a personalized training mode should be adopted according to their weaknesses. For nursing staff with low education level and poor clinical early warning ability, a counterpart assistance policy can be implemented by forming a group, in which nurses with strong clinical early warning ability and high education background are regarded as team leaders, forming a good learning atmosphere via each other's supervision. In addition, some scholars believed that although nursing staff's cognition of early warning ability of hospitalized patients was directly proportional to work experience and work years, the influence of these factors would not be very significant [18]. Researchers proposed that the experience of acute care of patients had no effects on nurses' risk assessment and decision-making ability under time pressure or task difficulty [19]. Nurses with rich clinical experience may not have strong nursing risk assessment and decision-making skills under time pressure or task difficulty [20]. Thus, we should focus on not only the learning of nurses' theoretical knowledge but also their ability to discern information and how to summarize and obtain valuable knowledge from past experience of failure or success in the future.

### 4.3. Nursing Staff Have a Strong Desire for Training on Early Warning Ability of Inpatients with “Three Infarcts and One Hemorrhage”

The results of this survey show that all the nurses surveyed believe that it is necessary to conduct training on the early warning ability of inpatients with “three infarcts and one hemorrhage,” indicating that nurses have a strong desire for risk warning knowledge training in Table 3. 47.14% of nurses think that it is better to train once a month, while 40.53% of nurses insist that the training frequency should be maintained once every six months. In this study, 61.37% of patients believe that the duration of each training should be kept at 0.5–1.0 h. For expected training mode and training location, 47.52% of nurses consider online self-study as the best approach, while 33.67% of nurses accept the training mode of face-to-face, centralized training in the department.

Risk early warning ability includes corresponding knowledge, skills, values, and attitudes, which is the basis of mastering nursing risk management skills and changing nursing risk management attitudes [21]. The previous research works have confirmed that the education and training of risk early warning were the key to enhance nurses' risk management ability, an important way to improve the effectiveness of nursing risk management, and an effective measure to solve safety issues of patients [22]. The training of risk early warning can not only effectively reduce the occurrence of adverse events but also improve patients' satisfaction and patient clinical outcomes and promote the quality of care. Previous researches reported that the construction of integrated medical-care risk management training system can effectively improve patients' satisfaction, reduce hospitalization time and complications, and improve the quality of care of nursing staff [23, 24]. Education and training can be carried out through a face-to-face approach, online learning mode, or distribution of learning materials related to risk early warning so that trainees can participate in the practice of a certain topic based on actual work experience, examples, and issues. The trainees will have an in-depth understanding of theoretical knowledge by these ways. The targeted, comprehensive, and diversified special training on the risk management ability of nurses at all levels can improve nurses' ability to identify potential risks and make proper responses in a timely manner. Intensified education and assessment of the risk early warning ability of patients with “three infarcts and one hemorrhage” for nursing staff can help form a long-term mechanism that can prevent and reduce the occurrence of nursing risks.

## 5. Conclusion

Nursing risk early warning ability is the first step of the nursing risk management process, which directly affects the accuracy of nursing risk assessment and the formulation of risk management decisions. Since nursing risks can be found everywhere in clinical medicine, the nursing risk early warning ability is particularly important. The ability of early warning and assessment of nursing risk turn the posttreatment of nursing risk events into preprevention, improving nurses' awareness of nursing safety incidents. In addition, it can help nurses identify the risks and unsafe factors in patients and greatly improve the quality and effectiveness of nursing works, while the study showed that the current status of nursing risk warning awareness and risk management ability in our hospital was not optimistic. Nursing staff in our hospital have a strong desire for training on early warning ability of inpatients with “three infarcts and one hemorrhage.” Diversified training mode and special training mode should be adopted according to the weakness of each nurse. The improvement of nursing risk management and emergency response ability will be the key research direction of nursing work in our hospital.

## Figures and Tables

**Figure 1:** The general information of the research object. (a) Gender, (b) education information, (c) professional title, (d) years of work, and (e) work location.

**Table 1:** Survey on the current status of nurses' risk warning knowledge of inpatients with “three infarcts and one hemorrhage” (*n* = 787).

Content item	*n* (%)	
	Yes	No
Professionally trained on the prevention and control of “three infarcts and one hemorrhage”	543 (69.00)	244 (31.00)
Had a good knowledge of cardiovascular risk factors	740 (94.03)	47 (5.97)
Acquired VTE risk assessment (Caprini score)	629 (79.92)	158 (20.08)
Aware of the Stroke Risk Scorecard	421 (53.49)	366 (46.51)
Experienced in the treatment of acute myocardial infarction	607 (77.13)	180 (22.87)
Had experience of treatment process of pulmonary embolism	529 (67.22)	258 (32.78)
Knew the treatment process of in-hospital stroke green channel	638 (81.07)	149 (18.93)
Had experience of first aid procedures for bleeding in hospital	546 (69.38)	241 (30.62)
Does the hospitalneed to increase knowledge related to “three infarcts and one hemorrhage”	745 (94.66)	42 (5.34)

*Note*. VTE: venous thromboembolism.

**Table 2:** Statistical investigation of selected nurses on the early warning ability of inpatients with “three infarcts and one hemorrhage” (*n* = 787).

Content item	Professionally trained on the prevention and control of “three infarcts and one hemorrhage”				Had a good knowledge of cardiovascular risk factors				Acquired VTE risk assessment (Caprini score)			
	Yes		No		Yes		No		Yes		No	
	*n*	%	*n*	%	*n*	%	*n*	%	*n*	%	*n*	%
Education background												
Junior college (*n* = 32)	17	53.12	15	46.88	28	87.50	4	12.50	26	81.25	6	18.75
Undergraduates (*n* = 605)	412	68.10	193	31.90	571	94.38	34	5.62	487	80.50	118	19.50
Masters and doctor (*n* = 150)	114	76	36	24	141	94	9	6.00	116	77.33	34	22.67

Professional title												
Junior professional (*n* = 368)	234	63.60	134	36.41	340	92.39	28	7.61	288	78.26	80	21.74
Intermediate professional (*n* = 306)	211	68.95	95	31.05	288	94.12	18	5.88	238	77.78	68	22.22
Deputy senior professional (*n* = 96)	84	87.50	12	12.50	95	98.96	1	1.04	86	89.58	10	10.42
Senior professional (*n* = 17)	14	82.35	3	17.65	17	100	0	0	17	100	0	0

Years of work												
≤2 (*n* = 85)	48	56.47	37	43.53	80	94.12	5	5.88	62	72.94	23	27.06
2–5 (*n* = 108)	70	64.81	38	35.19	96	88.89	12	11.11	82	75.93	26	24.07
5–10 (*n* = 239)	161	67.36	78	32.64	223	93.31	16	6.69	187	78.24	52	21.76
10–20 (*n* = 280)	201	71.79	79	28.21	267	95.36	13	4.64	231	82.50	49	17.50
＞20 (*n* = 75%)	63	84.00	12	16.00	74	98.67	1	1.33	67	89.33	8	10.67

Content item	Aware of the Stroke Risk Scorecard				Experienced in the treatment of acute myocardial infarction				Had experience of treatment process of pulmonary embolism			
	Yes		No		Yes		No		Yes		No	
	*n*	%	*n*	%	*n*	%	*n*	%	*n*	%	*n*	%

Education background												
Junior college (*n* = 32)	13	40.62	19	59.38	20	62.50	12	37.50	16	50.00	16	50.00
Undergraduates (*n* = 605)	319	52.73	286	47.27	460	76.03	145	23.97	396	65.45	209	34.55
Masters and doctor (*n* = 150)	89	59.33	61	40.67	127	84.67	23	15.33	117	78.00	33	22.00

Professional title												
Junior professional (*n* = 368)	184	50.00	184	50.00	264	71.74	104	28.26	219	59.51	149	40.49
Intermediate professional (*n* = 306)	162	52.94	144	47.06	242	79.08	64	20.92	215	70.26	91	29.74
Deputy senior professional (*n* = 96)	60	62.50	36	37.50	85	88.54	11	11.46	78	81.25	18	18.75
Senior professional (*n* = 17)	15	88.24	2	11.76	16	94.12	1	5.88	17	100.00	0	0.00

Years of work												
≤2 (*n* = 85)	37	43.53	48	56.47	61	71.76	24	28.24	50	58.82	35	41.18
2–5 (*n* = 108)	53	49.07	55	50.93	76	70.37	32	29.63	63	58.33	45	41.67
5–10 (*n* = 239)	128	53.56	111	46.44	177	74.06	62	25.94	150	62.76	189	79.08
10–20 (*n* = 280)	160	57.14	120	42.86	227	81.07	53	18.93	205	73.21	75	26.79
＞20 (*n* = 75%)	43	57.33	32	42.67	66	88.00	9	12.00	61	81.33	14	18.67

Content item	Knew the treatment process of in-hospital stroke green channel				Had experience in first aid procedures for bleeding in hospital				Does the hospital need to increase knowledge related to“ three infarcts and one hemorrhage”			
	Yes		No		Yes		No		Yes		No	
	*n*	%	*n*	%	*n*	%	*n*	%	*n*	%	*n*	%

Education background												
Junior college (*n* = 32)	26	81.25	6	18.75	20	62.50	12	37.50	26	81.25	6	18.75
Undergraduates (*n* = 605)	483	79.83	122	20.17	416	68.76	189	31.24	520	85.95	85	14.05
Masters and doctor (*n* = 150)	129	86.00	21	14.00	110	73.33	40	26.67	127	84.67	23	14.67

Professional title												
Junior professional (*n* = 368)	281	76.36	87	23.64	241	65.49	127	34.51	312	84.78	56	15.22
Intermediate professional (*n* = 306)	249	81.37	57	18.63	213	69.61	93	30.39	265	86.60	41	13.40
Deputy senior professional (*n* = 96)	92	95.83	4	4.17	76	79.17	20	20.83	83	86.46	13	13.54
Senior professional (*n* = 17)	16	94.12	1	5.88	16	94.12	1	5.88	13	76.47	3	17.65

Years of work												
≤2 (*n* = 85)	58	68.24	27	31.76	49	57.65	36	42.35	76	89.41	9	10.59
2–5 (*n* = 108)	81	75.00	25	23.15	69	63.89	39	36.11	91	84.26	17	15.74
5–10 (*n* = 239)	189	79.08	150	62.76	160	66.95	179	74.90	196	82.01	43	17.99
10–20 (*n* = 280)	238	85.00	42	15.00	208	74.29	72	25.71	247	88.21	33	11.79
＞20 (*n* = 75%)	72	96.00	3	4.00	60	80.00	15	20.00	63	84.00	12	16.00

**Table 3:** Nursing staff's needs for the early warning ability and related training of “three infarcts and one hemorrhage” inpatients (*n* = 787).

Content item	The number of approvers	The percentage of approvers
It is necessary to conductknowledge training-related “three infarcts and one hemorrhage” onnurses	787	100
Appropriate training frequency		
Once a week	34	4.32
Once a month	371	47.14
Once every six months	319	40.53
Once a year	63	8.01

The duration of each training		
0–0.5 h	188	23.89
0.5 h–1 h	483	61.37
1-2 h	102	12.96
2-3 h	14	1.78

Expected training mode and training location		
Onlineself-study	374	47.52
Face-to-face, centralized training indepartment	265	33.67
Face-to-face, centralized training inhospital	148	18.81

## Data Availability

The data used to support the findings of this study are available from the corresponding author upon request.
